# Regulatory Role of miRNAs and lncRNAs in Gout

This article has been retracted.

**DOI:** 10.1155/2022/6513565

**Published:** 2022-06-29

**Authors:** Jianlong Shu, Minhua Chen, Chunse Ya, Ruixia Yang, Fengzhen Li

**Affiliations:** ^1^Department of Rheumatology, Guangxi International Zhuang Medicine Hospital, Nanning, Guangxi, China 530201; ^2^Department of Ultrasound, Guangxi International Zhuang Medicine Hospital, Nanning, Guangxi, China 530201; ^3^Graduate School, Guangxi University of Chinese Medicine, Nanning, Guangxi, China 530201; ^4^Department of Cardiology, Guangxi International Zhuang Medicine Hospital, Nanning, Qiuyue Road No. 8, Liang Qing District, Nanning, Guangxi Zhuang Autonomous Region, China 530201

## Abstract

**Objective:**

To explore the regulatory functions of ceRNA networks in the nosogenesis of gout and search for potential therapeutic targets.

**Methods:**

We searched the GEO database and downloaded the lncRNA microarray chipset GSE160170. This matrix series was analyzed to yield differentially expressed lncRNAs and mRNAs. Then, the correlations between lncRNAs and miRNAs were obtained by comparing the highly conserved miRNA families. The predicted miRNA-regulating mRNAs were matched to the differentially expressed mRNAs from the chipset analyses to obtain miRNA–mRNA interactions. Next, we used the Cytoscape software to model ceRNA networks and the STRING database to determine their protein–protein interactions. The R software was used to algorithmically screen the functional pathways of key PPI modules in the ceRNA networks.

**Results:**

A total of 354 lncRNAs (140 downregulated and 214 upregulated) and 693 mRNAs (399 downregulated and 294 upregulated) were differentially expressed between the gout group and the healthy group. The ceRNA network of differentially expressed lncRNAs contained 86 lncRNAs (35 downregulated and 51 upregulated), 29 miRNAs, and 57 mRNAs. The processes identified in the GO enrichment analysis included gene transcription, RNA polymerase II transcription, and the regulation of cell growth and apoptosis. The pathways identified in the KEGG enrichment analysis included IL-17, TNF, and MAPK signaling. Nine lncRNAs (AC104024, AC084082, AC083843, FAM182A, AC022819, FAM215B, AP000525, TTTY10, and ZNF346-IT1), eleven miRNAs (hsa-miR-1297, hsa-miR-17-5p, hsa-miR-429, hsa-miR-139-5p, hsa-miR-449c-5p, hsa-miR-125a-5p, hsa-miR-125b-5p, hsa-miR-23b-3p, hsa-miR-217, hsa-miR-363-3p, and hsa-miR-20b-5p), and nine mRNAs (JUN, CASP2, PMAIP1, FOS, TNFAIP3, MAP3K8, BTG2, NR4A2, and DUSP2) were identified in the exploration of the key modules.

**Conclusion:**

Characterization of ceRNA networks could be a promising approach for better understanding the pathogenesis of gout, with the TTTY10/hsa-miR-139-5p/AP-1 axis likely to be of clinical significance.

## 1. Introduction

Gout, also known as arthritis rheumatica, is a disease characterized by the precipitation of monosodium urate crystals (MSU) in arthroses. Its prevalence varies worldwide, but the illness onset tends to occur in early adulthood [1]. In China, the incidence of gout ranges from 1% to 3%. Arthritic destruction and multiple organ involvement usually result from disease deterioration due to insufficient treatment [2]. Despite recent studies investigating the correlation of pathogenic physiology with disease progression, the underlying molecular mechanism remains unclear [3]. Our objective is to explore the nosogenesis of gout and discover potential biomarkers and therapeutic targets to support the development of new therapeutic strategies in this field.

Only 2% of human genes are eventually translated into functional proteins, while the rest are transcribed into so-called noncoding RNAs (ncRNAs) [4, 5]. It has been shown that these ncRNAs could regulate the expression of other genes. ncRNAs are classified as microRNAs (miRNAs) or long noncoding RNAs (lncRNAs) depending on their lengths. To explain the mechanisms by which ncRNAs modulate disease progression, it has been hypothesized that competing endogenous RNAs (ceRNAs) could emulate miRNAs, bind to a messenger RNA (mRNA), and prevent its translation [6, 7]. The miRNA response elements (MREs) of lncRNAs can also bind to mRNAs and compete with miRNAs [8]. RNA molecules transcribed by RNA polymerase II are longer than two hundred nucleotides and lack a reading frame are considered lncRNAs [9]. In gout, these molecules facilitate the degradation of the extracellular matrix in cartilage cells and transduce inflammatory signals. They can also mediate disease severity by regulating the invasion pathways of fibroblast-like synoviocytes [10, 11]. miRNAs regulate gene expression via subtle and intricate mechanisms. They have been shown to initiate inflammation in acute gout as essential constituents of MSU-induced inflammatory pathways [12, 13], with lncRNAs playing analogous roles in this process [3]. Although the involvement of ceRNAs in various disorders has been verified, few reports have demonstrated their roles in gout. Thus, this study was conceived to further investigate the interactions of three RNA subtypes (lncRNA, miRNA, and mRNA) in regulating gene transcription in gout.

## 2. Methods

### 2.1. Search Strategy

We obtained the relevant lncRNA microarray and expression data from the NCBI GEO database (https://www.ncbi.nlm.nih.gov/geo/) dating from January 2010 to March 2021 via searching using the following keywords: “Gout”, “lncRNA”, and “Human”.

### 2.2. Database Downloads

Based on the above results, the GSE160170 dataset (platform GPL21827, probe Agilent_079487, Arraystar human microarray V4; https://www.ncbi.nlm.nih.gov/geo/) was downloaded from the GEO database, including its matrix series and platform files. This chipset consisted of analyses of twelve peripheral blood samples, among which half were from healthy subjects and half from gout patients.

### 2.3. Reannotation and Comparison

The PERL software (Edition 5.30.0) was utilized to reassign the probe nucleotide sequences from the GEO platform into FASTA format. Next, the nucleotide sequences of all human transcribed sequences were downloaded from the GENCODE platform (https://www.gencodegenes.org/). They were compared with the probe sequences to yield probe files with corresponding gene labels.

### 2.4. Annotation of Matrix Series

To distinguish mRNAs from lncRNAs, the PERL software was applied to compare the matrix series to the probe files to match the probe IDs in the matrix series with the corresponding gene labels. Then, we used the downloaded human gene annotation file (.gtf file) to acquire the additional gene data in the software.

### 2.5. Expression Variation Analysis

We used the R software (Edition 4.0.4, “limma” mode) to analyze the differentially expressed genes in the matrix series. Using the setting logFC (log2 − fold change) > 1 or < -1 along with adjusted *P* value < 0.05 as the prerequisite parameters, a volcano plot was mapped following the differential lncRNAs and mRNAs from the chipset. The HETML software was then used to generate dendrograms and heat maps of hierarchical clustering. In the plots, LogFC > 1 and LogFC < 1 indicated the upregulation and downregulation of this particular differential lncRNA in gout patients, respectively.

### 2.6. Prediction of miRNA Binding to lncRNAs

We downloaded the conserved miRNA family files from the miRcode platform (http://www.mircode.org/). Then, the PERL software was used to verify the interactions between differentially expressed lncRNAs and miRNAs to predict their connections.

### 2.7. Prediction of mRNAs Regulated by miRNAs

The predictions of regulatory relationships between mRNA and miRNAs were made based on the miRDB database (http://mirdb.org/), the miRTarBase database (http://mirtarbase.mbc.nctu.edu.tw/php/index.php), and the TargetScan database (http://www.targetscan. org/vert_72/). Only those pairs predicted by all three databases were retained for further study. The PERL software validated the sequence identity when the prediction results were compared with the differential mRNAs from the chipset and thus yielded a set of miRNA–mRNA associations.

### 2.8. Construction of ceRNA Networks

We modeled coexpressed lncRNA–miRNA–mRNA triads according to the ceRNA concept. The ceRNA networks of upregulated and downregulated differentially expressed lncRNAs were plotted by Cytoscape software (Edition 3.8.2). The connection between the two frame points represented a regulatory relationship.

### 2.9. Construction and Analysis of the Protein–Protein Interaction (PPI) Network

We enacted a confidence interval > 0.9 as the parameter to screen protein components in the PPI network and evaluated their interactions by searching the STRING database (Edition 11.0, https://string-db.org/). The Cytoscape software delineated the network plot after loading in the STRING database. Next, using the setting degree cutoff = 2, score cutoff = 0.2, k − core = 2, and max.depth = 100 as the parameters, we visualized the essential lncRNA–miRNA–mRNA subnetworks by using the algorithms in the MCODE plugin. The GO and KEGG pathway annotations of every key lncRNA were further identified by assessing the original and subnetwork mRNAs in the ceRNA networks.

### 2.10. GO and KEGG Enrichment Analysis

To determine the functions of the key PPI modules, the DAVID database was filtered for GO enrichment analysis. The gene data were then exported into Excel, and the GO enrichment analysis plot was made by GraphPad Prism (Edition 9.0.2). We also used the R software to perform KEGG enrichment analysis and assay the relevant pathways. *P* value < 0.05 represented statistical significance.

### 2.11. Exploration of the Key ceRNA Networks

The analysis of miRNAs competitively bound to lncRNAs and mRNAs was performed by exploring the KEGG-enriched mRNAs in the ceRNA networks. The key ceRNA network was generated from the above results in the Cytoscape software to search for pathways regulating crucial genes in the KEGG enrichment analysis plot.

## 3. Results

### 3.1. Differentially Expressed lncRNAs and mRNAs

A total of 354 differentially expressed lncRNAs were identified by comparing the gout group and the healthy group by setting ∣logFC | >1 and adjusted *P* value < 0.05 as the parameters. A total of 140 were downregulated, whereas the rest were upregulated. A total of 693 mRNAs were identified via similar comparisons, among which 399 were downregulated and 294 were upregulated.  Figure 1 shows the volcano plot of hierarchical clustering of differentially expressed lncRNAs.  Figure 2 shows the dendrogram and heat map of hierarchical clustering of differentially expressed lncRNAs, and Figure 3 shows the dendrogram and heat map of hierarchical clustering of differentially expressed mRNAs.

### 3.2. The ceRNA Network of Differentially Expressed lncRNAs

There were 86 lncRNAs in the ceRNA network (35 were downregulated, 51 were upregulated). Twenty-nine miRNAs were screened out by the predictions of all three databases (miRDB, miRTarBase, and TargetScan). The mRNAs regulated by those miRNAs were further compared with those from the chipset data, and we obtained 57 common mRNAs. Figures 4 and 5 show the ceRNA networks of upregulated and downregulated differentially expressed lncRNAs.  Table 1 lists the upregulated and downregulated mRNAs in the ceRNA network.

### 3.3. Analyses of the PPI Network and Key Modes

Using the setting confidence coefficient > 0.4, 33 protein–protein interactions involving 57 proteins were obtained. Two key modules of protein–protein interactions were identified by the Cytoscape MCODE mode. Module 1 consisted of JUN, CASP2, and PMAIP1. Module 2 consisted of FOS, TNFAIP3, MAP3K8, BTG2, NR4A2, and DUSP2 (Figure 6).

### 3.4. GO Enrichment Analysis

Given a *P* value < 0.05, we identified 57 mRNAs for GO enrichment analysis. These subjects included numerous cellular components, biological process, and molecular function terms. The enriched biological process terms included DNA transcription, cell proliferation, RNA polymerase II promoter transcription, cell program death, lipopolysaccharide metabolism, cell maturation, mitosis, bone mineralization, neuron programmed cell death, and stress responses. The enriched cellular component terms were nuclei, cytoplasm, and lipids. Their enriched molecular function terms were protein binding, transcription factor activities, and sequence-specific DNA binding responsible for modulating RNA polymerase II promoters and distant enhancers. We also evaluated the nine key modules in the GO enrichment analysis. Similarly, these processes included neuronal program death regulation, cell maturation, the reaction to extracellular stimulus, pri-miRNA transcription of RNA polymerase II, regulation of the activities of sequence-specific DNA transcription factors, cellular responses to hormones, cytokines and mechanical stimuli, signal conduction of SMAD protein, DNA damage signaling, and transforming growth factor (TGF) receptor signaling pathways. These modules were responsible for regulating the production of nuclear and cytoplasmic materials and facilitating protein and DNA associations, the activities of protein heterodimers and transcription factors, the binding of sequence-specific DNAs and R-SMADs, and other processes (Figure 7).

### 3.5. KEGG Enrichment Analysis

We set the *P* value < 0.05 to analyze the pathways involving TNF, IL-17, and MAPK signaling via the “Colorspace,” “Stringi,” and “BiocManager” modes in R software. The outcomes are shown in Figure 8.

### 3.6. Key ceRNA Network

The key ceRNA network was filtered to identify the key modules in which lncRNAs are bound to miRNAs in competition with the enriched mRNAs. We discovered that the extents of up- and downregulation were identical in the same groups of mRNAs and miRNAs. The eleven miRNAs identified to be under the influences of their respective lncRNAs were as follows: hsa-miR-1297, hsa-miR-17-5p, hsa-miR-429, hsa-miR-139-5p, hsa-miR-449c-5p, hsa-miR-125a-5p, hsa-miR-125b-5p, hsa-miR-23b-3p, hsa-miR-217, hsa-miR-363-3p, and hsa-miR-20b-5p (Figures 9 and 10).

### 3.7. Key Regulatory Network

Considering the identification of the TNF and IL-17 signaling pathways in the KEGG enrichment analysis, the FOS and JUN mRNA components were likely to act as the principal factors in the pathophysiology of gout (https://www.kegg.jp/pathway/map04657, https://www.kegg.jp/pathway/map04668). They bounded to hsa-miR-139-5P in competition with lncRNAs including AC104024, AC084082, AC083843, FAM182A, AC022819, FAM215B, AP000525, TTTY10, and ZNF346-IT1. Among them, AC104024, AC084082, AC083843, and FAM182A were downregulated, and AC022819, FAM215B, TTTY10, and ZNF346-IT1 were upregulated (Table 2). We constructed the representative ceRNA signaling pathways in gout based on the aforementioned results using the pathway tool software Edition 2.0 (Figure 11).

## 4. Discussion

Gout, a type of arthritis caused by the precipitation of MSU crystals in joints, can result in acute inflammation and damage to adjacent tissues. Its representative features are the rapid onset of sharp pain and self-limiting symptoms (lasting 3-14 days) [14]. Moreover, its incidence is increasing in developed countries [15]. Common comorbidities include cardiovascular diseases, nephrolithiasis, obesity, and diabetes. In addition to the physical pain it causes for patients, medical treatments for gout are often unaffordable, and this disease impacts the productivity of society as a whole [16]. The scientific consensus is that the physiological basis of gout involves the activation of the NF-KB pathways by Toll receptors after MSU crystals are recognized by macrophages [17]. This response releases IL-1*β* from inflammasomes via the NLRP3 signaling to generate rheumatic manifestations [18]. Inflammatory signals recruit neutrophils to capture MSU by exocytosing extracellular traps; then, macrophages engulf apoptotic neutrophils to relieve inflammation. This mechanism may explain the self-limiting symptoms of the disease [19].

As the crucial roles of ceRNAs in inflammatory disorders are well accepted, studies have increasingly emphasized the strong correlations between gout and inflammatory mediators such as the IL-1*β*, TNF-*α*, and NLRP3 inflammasomes [20]. Early evidence attributed the disease to mutations in protein-coding genes. However, the study of noncoding RNAs revealed that the mutations in lncRNAs, the occupancy of which was 98% in the transcription group, might account for illness onset. Moreover, lncRNAs are considered good biomarkers and targets for clinical diagnosis, prognosis, and pharmaceutical manufacture [21–23]. An increasing number of miRNAs and lncRNAs were discovered to be involved in regulating gout [24]. Aberrant expression of miRNAs in MSU-induced macrophages and joints triggers the production of cytokines as proinflammatory factors [25]. Various studies have shown that such specific expression of lncRNAs in T and B cells implies that they are regulators of immune cells to modulate inflammation in gout [26, 27]. Further analyses of relevant miRNAs/lncRNAs showed that they supervised inflammatory processes via the MAPK, NF-KB, PI3K/AKT, NLRP3, and TLR pathways [28].

Our study indicated that the differentially expressed genes in gout, such as Act1, TRAF6, NF-*κ*B, AP-1, FOS, JUN, IL-1*β*, and COX-2, were mainly involved in the IL-17 and TNF signaling pathways. The FOS and JUN genes were differentially expressed after matching with the mRNAs in the key ceRNA network. Nine lncRNAs that could bind competitively to hsa-miR-139-5P, the potential miRNA target to which the FOS and JUNE genes are also bound, were identified. Among these lncRNAs, AC104024, AC084082, AC083843, and FAM182A were downregulated, whereas AC022819, FAM215B, AP000525, TTTY10, and ZNF346-IT1 were upregulated. Intriguingly, both upregulation and downregulation were observed in AC083843 and FAM182A.

Act1, one of the downstream components of the IL-17 pathway, was shown to stabilize mRNA expression and mediate inflammatory signal conduction as an adaptor of the IL-17 receptor [28]. TRAF6, another downstream component, acts as the receptor kinase of IL-17 to trigger signal transmission through the pathway by inducing NF-KB to activate inflammatory factors and cytokines (NF-KB and AP-1 are mutually dependent). AP-1 exhibits paradoxical properties in the regulation of gene transcription. Its subunits include c-Fos, c-Jun, Jun B, and Jun D, of which c-Fos and c-Jun shared the most extensive transcription initiation activities. Many AP-1 binding sites have been reported to exist in the promoters of inflammatory factors (IL-1*β* and TNF-*α*), growth factors, and matrix metalloproteinase (MMP2 and MMP9) [29–31]. They alternate between proinflammatory and prophagocytic processes [29]. Nevertheless, some AP-1 downstream targets inhibit inflammatory responses, such as the Th2 cytokines IL-4, IL-5, and IL-13, whose expression is subject to regulation by AP-1 through its binding to the corresponding gene promoters [32]. In the IL-17 signaling pathway, the subtypes IL-17A, IL-17B, IL-17C, and IL-17F are proinflammatory, whereas IL-17E acts as an anti-inflammatory agent. COX-2 is another gene under the regulation of AP-1. Its localization on the nuclear surface allows convenient entrance into the nucleus and direct influence on gene expression. The promoter of the COX-2 gene contains multiple TF binding sites, including those for AP-1 and NF-KB [33]. PGE2, one of the essential products of COX-2, enhances the local inflammatory response and recruits circulating leukocytes to secrete cytokines [34].

Several studies have reported on the activities of miR-139-5p, an miRNA that binds to the JUN and FOS genes [35]. Analysis using the DIANA TOOLS software (http://diana.imis.athena-innovation.gr/DianaTools/index.php) confirmed the binding sites for miR-139-5p within JUN and TRAF6. Recent publications have indicated that miR-139-5p decreases the plasma concentrations of IL-1*β* and TNF-*α* by adjusting TRAF6 to alter the inflammatory and oxidizing responses of macrophages. Furthermore, miR-139-5p was shown to promote the activities of T cells by targeting c-Jun and c-Fos [36]. Therefore, we speculated that miR-139-5p might be critically important in the nosogenesis of gout.

Among the lncRNAs competing with miR-139-5p, FAM182A had the most extensive downregulation, while TTTY10 was the most upregulated. Although the functions of lncRNAs other than TTTY10 are yet to be explored, nine other lncRNA subjects were hypothesized to produce similar effects. TTTY10 participates in cell attachment, transcription, signal conduction, growth, and differentiation via the FoxO1 gene [37]. It is a crucial transcription factor that shares identical regulatory functions with NF-KB and AP-1. FoxO1 can also relieve inflammation by inhibiting the NF-KB-, FoxO1-, and AP-1-related pathways [38, 39]. Thus, we concluded that TTTY10 was of great importance in executing the inflammatory responses of immune cells.

Due to the involvement of IL-17 in immune regulatory functions, the effects of IL-17 inhibitors have been investigated in autoimmune diseases. The US Food and Drug Administration (FDA) has approved the IL-17 inhibiting monoclonal antibody secukinumab (trade name: Cosentyx) to treat severe plaque psoriasis [40]. Further, the anti-IL-23 antibody ustekinumab was shown to effectively treat moderate-to-severe psoriasis by indirectly reducing IL-17 [41]. Presently, TNF-*α* inhibitors such as infliximab, adalimumab, etanercept, certolizumab pegol, and golimumab are being clinically used to treat inflammatory diseases [42–44]. In a case report by Zhang et al., the researchers showed that the TNF-*α* antagonist etanercept, given at 25 mg subcutaneous injection two times a week, could significantly relieve joint pain one day after treatment and completely relieve it after five days of treatment. Further, after 2 weeks, the levels of C-reaction protein (CRP) and blood routine examination returned to normal [44]. In a genome-wide study by White et al., the authors showed the promising effects of certolizumab pegol in moderate to severe rheumatoid arthritis [45].

Lastly, although lncRNAs may participate in the progression of arthritis by competing with miRNAs, few studies have reported the existence of binding sites between the aforementioned lncRNAs and miR-139-5p; therefore, no sufficient evidence supports the hypothesis that lncRNAs regulate cytokine secretion via miR-139-5p. We designed this study in the hope of adding new knowledge to the currently available options for gout therapy. The power of our research, however, had some limitations given the predictive nature of bioinformatics analyses and several clinical trials. No systemic proof has been found beyond the existence of these lncRNA–miRNA–mRNA networks. In future work, we expect to verify the differential expression of lncRNAs in patients and healthy subjects in the clinic. The principle will be to study the regulatory mechanisms of lncRNAs binding to miR-139-5p in competition with the JUN and FOS genes. The mechanisms underlying the interactions between the subtypes of c-fos and c-jun, as well as how lncRNAs and miR-139-5p restrict their transcription, require further detailed characterization.

In conclusion, the principle of targeting miRNAs and lncRNAs in gout therapy urges more prospective explorations in the clinic.

## Figures and Tables

**Figure 1:** Volcano plot of hierarchical clustering of differentially expressed lncRNAs (red: upregulated lncRNAs, green: downregulated lncRNAs).

**Figure 2:** Dendrogram and heat map of hierarchical clustering of differentially expressed lncRNAs. Note: the *x*-axis shows the sample names of the chipsets. The *y*-axis is labeled with the names of lncRNAs. Red represents a high level of relative expression; green represents a low relative expression level. Black indicates nonsignificant differences in relative expression. Blue represents peripheral blood samples from healthy subjects; pink represents peripheral blood samples from gout subjects. The branches on the *y*-axis represent the clustering of various lncRNAs. The twelve lncRNA samples were clustered into three categories sharing similar differential expression patterns.

**Figure 3:** Dendrogram and heat map of hierarchical clustering of differentially expressed mRNAs. Note: the *x*-axis shows the sample names of the chipsets. The *y*-axis is labeled with the names of mRNAs. Red indicates a high level of relative expression; green indicates a low relative expression level. Black indicates nonsignificant differences in relative expression. Blue represents peripheral blood samples from healthy subjects; pink represents peripheral blood samples from gout subjects. The branches on the *y*-axis represent the clustering of various lncRNAs. The twelve mRNA samples were clustered into two categories sharing similar differential expression patterns.

**Figure 4:** The ceRNA network of upregulated lncRNAs. Note: orange represents miRNAs. Purple represents lncRNAs. Green represents mRNAs. The connections between items represent their regulatory relationships.

**Figure 5:** The ceRNA network of downregulated lncRNAs. Note: orange represents miRNAs. Purple represents lncRNAs. Green represents mRNAs. The connections between items represent their regulatory relationships.

**Figure 6:** Protein–protein interaction network. Note: the connections between items represent protein–protein interactions. Two key modules were identified by Cytoscape MCODE mode. Orange represents the subjects in module 1; green represents the subjects in module 2.

**Figure 7:** GO enrichment analyses.

**Figure 8:** KEGG enrichment analysis.

**Figure 9:** The ceRNA networks of upregulated lncRNAs.

**Figure 10:** The ceRNA networks of downregulated lncRNAs.

**Figure 11:** Representative signaling pathways of ceRNAs in gout.

**Table 1:** Downregulated and upregulated mRNAs in ceRNA networks.

mRNA	Genes
Downregulated mRNAs	NR4A2, CADM2, FYCO1, SLX4, ADM, MCC, BACH2, BTG2, ZNF217, VCPIP1, ZBTB10, TXNIP, KLF10, LMLN, UTRN, KIF13A, BTG1, SSH2, STK11, MTSS1, SACS, NCOA5, C9orf72, YRDC, MAP3K8, BOD1, CAPN15, TIPARP, PMAIP1, BTG3, C9orf40, GATA2, TNFAIP3, FNIP1, INPP5A, HMGB3, SCML2, JUN, TUBB2A, TSC22D2, NUP43, PLAG1, BRWD1, STARD13, QSER1, FBXO48, RNF145, DUSP2, IPO7, ARMC1, FOS, UBE3C, PTGS2, CASP2, RAP1B, AXIN2, LRRC2
Upregulated mRNAs	RAP1B, BOD1, TUBB2A, FBXO48, AXIN2, TNFAIP3, JUN, CASP2, ZBTB10, INPP5A, BRWD1, BTG3, MAP3K8, DUSP2, TSC22D2, GATA2, MCC, SCML2, KLF10, ADM, LMLN, BACH2, ZNF217, CAPN15, KIF13A, FYCO1, FNIP1, STK11, BTG2, UBE3C, SACS, BTG1, SLX4, STARD13, MTSS1, NR4A2, CADM2, LRRC2, RNF145, C9orf40, NUP43, QSER1, TXNIP, SSH2, PTGS2, TIPARP, NCOA5, UTRN, HMGB3, PLAG1, ARMC1, VCPIP1, IPO7, C9orf72, PMAIP1, FOS, YRDC

**Table 2:** Parameters of up- and downregulated lncRNAs.

lncRNA	logFC	AveExpr	*t*	*P* value	Adjusted *P* value
TTTY10	1.182591	4.3677	5.798418	0.000112	0.001618
AC022819	1.109496	3.124482	10.29479	4.81E-07	4.05E-05
FAM215B	1.071295	4.445856	4.068199	0.001797	0.011922
ZNF346-IT1	1.042113	6.191628	8.010408	5.82E-06	0.000217
AP000525	1.02872	9.056032	3.880768	0.002485	0.01497
AC084082	-1.0971	3.392878	-4.0296	0.00192	0.012499
AC083843	-1.12263	6.323656	-4.40739	0.00101	0.007905
AC104024	-1.22902	4.098741	-5.29094	0.000242	0.002786
FAM182A	-1.3358	3.573437	-4.38903	0.001042	0.008078

Note: logFC > 1 indicates upregulation, logFC < −1 indicates downregulation.

## Data Availability

The data used to support the findings of this study are available from the corresponding author upon request.
